# miR‐30d‐5p suppresses proliferation and autophagy by targeting ATG5 in renal cell carcinoma

This article has been retracted.

**DOI:** 10.1002/2211-5463.13025

**Published:** 2020-12-19

**Authors:** Liang Liang, Zheng Yang, Qian Deng, Yazhuo Jiang, Yongyi Cheng, Yi Sun, Lei Li

**Affiliations:** ^1^ Department of Urology The First Affiliated Hospital of Xi'an Jiaotong University China; ^2^ Medical College of Xi'an Jiao Tong University China; ^3^ Department of Urology Shaanxi Provincial People's Hospital Xi'an China; ^4^ Department of Urology The Third Affiliated Hospital of Xi'an Jiaotong University China

**Keywords:** ATG5, autophagy, miR‐30d‐5p, proliferation, renal cell carcinoma

## Abstract

Previous reports have shown that miR‐30d‐5p functions as a tumor suppressor in prostate cancer and gallbladder carcinoma, but its role in renal cell carcinoma (RCC) remains elusive. This study was designed to explore the functional role of miR‐30d‐5p in proliferation and autophagy of RCC. Our results show that miR‐30d‐5p is significantly down‐regulated in RCC tissues compared with normal tissues. miR‐30d‐5p overexpression suppressed cell proliferation, cell‐cycle G1/S transition and autophagy, but promoted apoptosis in RCC cell lines (786‐O and ACHN). Intriguingly, autophagy‐related gene 5 (ATG5) was directly targeted by miR‐30d‐5p, as shown using luciferase reporter assay and biotin‐avidin pull‐down assay. Moreover, overexpression of ATG5 attenuated the inhibitory effect of miR‐30d‐5p on proliferation and autophagy in 786‐O cells. These results suggest that miR‐30d‐5p suppresses proliferation and autophagy in RCC cells by targeting ATG5, and this pathway may be a suitable basis for the design of novel cancer therapeutics.

## Graphical abstract

miR‐30d‐5p suppresses cell proliferation, G1/S transition and autophagy, and promotes apoptosis by targeting autophagy‐related gene 5 in renal cell carcinoma.

**Abbreviations**
ATG5: autophagy‐related gene 5
CCK‐8: Cell Counting Kit‐8
MUT: mutant
NC: negative control
PI: propidium iodide
qRT‐PCR: quantitative RT‐PCR
RCC: renal cell carcinoma
SD: standard deviation
WT: wild‐type

Renal cell carcinoma (RCC), including two main histological subtypes (clear cell RCC and papillary RCC) [1], is the third leading cause of urological malignancies, accounting for ~3% of all adult malignancies [2]. Despite great efforts having been made in multimodal approaches and strategies, the prognosis of patients with RCC still remains unsatisfactory [3, 4. Therefore, it is urgently imperative to investigate the molecular mechanisms underlying the pathogenesis of RCC to improve treatment and prognosis for patients with RCC.

MicroRNAs (miRNAs/miRs), a group of small noncoding RNAs ~22–24 nucleotides in length, have been widely reported to negatively regulate their target genes at the posttranscriptional level by binding to the 3′ UTR of target mRNAs, which play an important regulatory role in diverse cellular processes, including proliferation, apoptosis and autophagy [5, 6, 7. Accumulating evidence indicates that miRNAs are aberrantly expressed in the development and progression of cancers by acting as tumor suppressors or oncogenes [8, 9, 10. Recently, miR‐30d‐5p has been demonstrated to participate in tumor development by functioning as a tumor suppressor. For example, miR‐30d‐5p significantly inhibits the growth and motility of non‐small cell lung cancer cells by directly targeting cyclin E2 [11]. He *et al*. [12] showed that miR‐30d‐5p suppressed the aggressive progression of gallbladder carcinoma by targeting lactate dehydrogenase‐A. Similarly, Song *et al*. [13] reported the tumor‐suppressive function of miR‐30d‐5p in prostate cancer cell proliferation and migration by targeting NT5E. However, there are no reports on the expression and biological functions of miR‐30d‐5p in RCC progression.

Autophagy is a complex homeostatic process by inducing lysosomal degradation of damaged organelles and molecules to recycle metabolic substances for survival under adverse conditions [14]. Currently, the role of autophagy in tumor progression remains controversial. Degenhardt *et al*. [15] have reported the oncogenic autophagy in tumor cell survival. Conversely, autophagy could protect cells from oxidative stress and genomic instability in the early stages of cancer [16]. In RCC, Yuan *et al*. [17] demonstrated that mitochondrial E ubiquitin ligase 1 could promote autophagy to suppress the development of this disease, whereas Chow *et al*. [18] showed that autophagy suppression was associated with enhanced cytotoxicity induced by the covalent CDK7 inhibitor THZ1. Our previous bioinformatics prediction indicated that autophagy‐related gene 5 (ATG5) was a target gene of miR‐30d‐5p. Interestingly, the regulator function of miR‐30d‐5p in autophagy in different diseases has been illustrated as follows: increase of miR‐30d‐5p resulted in reduction of autophagy and increase of apoptosis in rat brains after hypoxic–ischemic injury [19]. miR‐30d‐5p was reported to decrease cell autophagy by targeting glycine decarboxylase to suppress hepatocellular carcinoma progression [20]. Nevertheless, whether miR‐30d‐5p played an important role in regulating cell proliferation and autophagy by targeting ATG5 in RCC has not been reported yet.

In this study, we first analyzed the expression of miR‐30d‐5p in RCC tissues and cell lines. Next, the functional roles of miR‐30d‐5p in cell proliferation, cell‐cycle progression, apoptosis and autophagy were investigated in RCC cells. Moreover, we explored whether ATG5 was a direct downstream regulator involved in miR‐30d‐5p regulating biological functions. Altogether, our findings may provide new insights into the treatment of RCC.

## Materials and methods

### Tissue collection

A total of 25 paired tumor tissues and matched adjacent tissues as normal tissues were surgically collected from patients with RCC at The First Affiliated Hospital of Xi'an Jiaotong University (Xi'an City, Shanxi, China); the tissues were immediately snap frozen in liquid nitrogen for subsequent use. The basic clinicopathological features are listed in Table 1. None of the patients had received any chemotherapy or radiotherapy. The written informed consent was signed by each patient. This study was conducted in accordance with the Declaration of Helsinki and with approval from the Ethics Committee of The First Affiliated Hospital of Xi'an Jiaotong University.

**Table 1:** The baseline characteristics of patients with RCC.

Characteristics	Cases (*n* = 25)
Sex	
Male	17
Female	8
Age, yr	
<60	12
≥60	13
Tumor size, cm	
<5	20
≥5	5
Histological type	
Clear cell	22
Papillary	3
TNM stage	
I–II	19
III–IV	6
Lymph node metastasis	
Negative	21
Positive	4

### Cell culture

Human RCC cell lines (786‐O, ACHN and Caki‐1) and normal kidney cell line HK‐2 were purchased from the American Type Culture Collection (Manassas, VA, USA). 786‐O cells were maintained in RPMI‐1640 media containing 10% FBS (Gibco, Thermo Fisher Scientific, Inc., Waltham, MA, USA). The other three cell lines were cultured in Dulbecco's modified Eagle’s medium supplemented with 10% FBS (Gibco). All cells were cultured and maintained at 37 °C in a humidified incubator with 5% CO_2_.

### Cell transfection

The miR‐30d‐5p mimics and negative control (miR‐NC) were chemically synthesized by GenePharma Co., Ltd. (Shanghai, China). The full‐length ATG5 ORF was cloned into vector pcDNA3.1(+) and named pcDNA3.1‐ATG5. For miR‐30d‐5p overexpression, 786‐O and ACHN cells were transfected with miR‐30d‐5p mimics when cells reached 70–80% confluence. In the rescue experiments, pcDNA3.1‐ATG5 or empty pcDNA3.1 plasmid was transfected into miR‐30d‐5p mimics or miR‐NC‐transfected 786‐O cells. The earlier transfection protocols were performed for 48 h using Lipofectamine 2000 reagent (Invitrogen, Carlsbad, CA, USA) following the manufacturer's instructions.

### Quantitative RT‐PCR

We first extracted all RNA with TRIzol reagent (Takara Biotechnology Co., Ltd.) and performed reverse transcription using TaqMan miRNA Reverse Transcription Kit (Thermo Fisher Scientific) or PrimeScript™ RT reagent kit (Takara Biotechnology Co., Ltd.) according to the manufacturer's instructions. With the SYBR Green qPCR SuperMix (Invitrogen), the expression levels of miR‐30d‐5p and ATG5 mRNA were determined on an ABI 7500 PCR System according to the thermocycling conditions: 50 °C for 2 min and 94 °C for 2 min, followed by 40 cycles of 94 °C for 15 s and 60 °C for 32 s. The primer sequences used for PCR were as follows: miR‐30d‐5p forward, 5′‐CCTGTTGGTGCACTTCCTAC‐3′ and reverse, 5′‐TGCAGTAGTTCTCCAGCTGC‐3′; U6 forward, 5′‐ATGACGTCTGCCTTGGAGAAC‐3′ and reverse, 5′‐TCAGTGTGCTACGGAGTTCAG‐3′; ATG5 forward, 5′‐AAAGATGTGCTTCGAGATGTGT‐3′ and reverse, 5′‐CACTTTGTCAGTTACCAACGTCA‐3′; GAPDH forward, 5′‐TGAACGGGAAGCTCACTGG‐3′ and reverse, 5′‐TCCACCACCCTGTTGCTGTA‐3′. The relative gene expression levels were calculated using the $2^{‐\Delta \Delta C_{t}}$method with U6 or GAPDH as the endogenous control.

### Cell proliferation assay

We used Cell Counting Kit‐8 (CCK‐8; Beyotime, Shanghai, China) to determine the cell proliferation ability in RCC cells. In brief, transfected cells were plated onto 96‐well plates at an initial density of 3 × 10^3^ cells per well. At 0, 24, 48, 72 and 96 h, each well was incubated with 10 μL CCK‐8 reagent for another 2 h at 37 °C. The proliferation ability was assessed by measuring the optical density value at a wavelength of 450 nm under a microplate reader.

### Flow cytometry assay

Flow cytometry assay was conducted to evaluate cell‐cycle distribution and apoptosis in transfected RCC cells. In brief, cells were seeded in 6‐cm dishes at a density of 2 × 10^5^ cells per well and cultured overnight. The next day, cells were harvested and fixed in 70% ice‐cold ethanol overnight at 4 °C. After being washed with PBS, cells were incubated with propidium iodide (PI) (Sigma‐Aldrich, St. Louis, MO, USA) for 15 min in the dark for cell‐cycle analysis. For apoptotic assay, cells were incubated with Annexin V–FITC and PI (Abcam, Cambridge, MA, USA) in the dark for 15 min. Afterward, stained cells were analyzed for cell‐cycle distribution, or apoptotic rate by the distribution and apoptosis of each phase of the cell cycle were measured by FACSCalibur flow cytometer (BD Biosciences, San Jose, CA, USA).

### Immunofluorescence assay

The expression of LC3B was observed by performing immunofluorescence assay. In brief, transfected cells were grown on glass coverslips overnight and fixed with 4% paraformaldehyde. After treatment with 0.2% Triton X‐100, cells were blocked with 2% BSA and incubated with primary antibody against LC3B (#ab48394, 1 : 200; Abcam) at 4 °C overnight, followed by staining with a fluorescent secondary antibody for 1 h. Finally, cell nuclei were stained with 0.2 mg·mL^−1^ 4′,6‐diamidino‐2‐phenylindole (DAPI) for 15 min and imaged with a fluorescence microscope (Olympus, Tokyo, Japan).

### Luciferase reporter assay

According to predicted results by TargetScan (http://www.targetscan.org/vert_71/), luciferase reporter assay was performed to confirm the binding sites between miR‐30d‐5p and ATG5 3ʹ UTR. In brief, the human 3′ UTR of ATG5 (UGUUUAC) containing the miR‐30d‐5p putative wild‐type (WT) binding sites or corresponding mutant (MUT) sites was cloned into the pGL3 luciferase reporter vector (Promega Corporation, Madison, WI, USA), which were named as WT‐ATG5 and MUT‐ATG5, respectively. Next, 786‐O or ACHN cells were plated (5 × 10^4^ per well) in 24‐well plates and transfected with miR‐30d‐5p mimics or miR‐NC together with WT‐ATG5 or MUT‐ATG5 using Lipofectamine 2000 reagent. At 48 h after transfection, relative luciferase activity was measured using a Luciferase reporter assay kit (Promega Corporation) with Renilla luciferase activity as an internal control.

### Western blot analysis

Transfected cells were lysed with radioimmunoprecipitation assay (RIPA) lysis buffer to extract all proteins, and the corresponding concentration was determined with BCA assay (Thermo Fisher Scientific, Inc.). Protein samples (30 µg) were resolved on 12% SDS/PAGE and electrotransferred onto poly(vinylidene difluoride) membranes. Afterward, the membranes were blocked with 5% skimmed milk for 2 h at room temperature and incubated with primary antibodies against LC3B (#ab48394, 1 : 500; Abcam), p62 (#ab56416, 1 : 500; Abcam), ATG5 (#ab108327, 1 : 500; Abcam), p21, Bad and β‐actin (cat. no. 4970; 1 : 1000; Cell Signaling Technology, Inc., Danvers, MA, USA) overnight at 4 °C. After being washed twice with PBS, the membranes were incubated with horseradish peroxidase‐conjugated secondary antibodies for 2 h at room temperature. The protein bands were visualized with enhanced chemiluminescence (Thermo Scientific, Rockford, IL, USA).

### Biotin‐avidin pull‐down assay

Biotinylated WT miR‐30d‐5p (miR‐30d‐5p‐Bio), MUT miR‐30d‐5p (miR‐30d‐5p‐MUT‐Bio) or NC (NC‐Bio) was obtained using the Biotin RNA Labeling Mix (GenePharma Co., Ltd), which were respectively transfected into 786‐O or ACHN cells for 48 h. Then, the cells were incubated with magnetic beads for 1 h at room temperature. After treatment with washing buffer, the bound RNAs were obtained and analyzed by quantitative RT‐PCR (qRT‐PCR).

### Statistical analysis

All quantitative experiments were performed three times, and data are presented as the mean ± standard deviation (SD). We evaluated the statistical differences with paired Student's *t*‐test or ANOVA followed by Tukey's *post hoc* test or Dunnett's multiple comparisons test. The expression correlation between miR‐30d‐5p and ATG5 in tumor tissues was analyzed using Pearson's correlation test. The threshold for statistical significance was set at *P* < 0.05.

## Results

### miR‐30d‐5p was significantly down‐regulated in RCC

To investigate whether miR‐30d‐5p played an important role in the progression of RCC, we first sought to know the level of miR‐30d‐5p in 25 paired RCC tissues and adjacent normal tissues. Statistical analysis (Fig. 1A) and single values (Fig. 1B) of miR‐30d‐5p from qRT‐PCR analysis consistently showed that miR‐30d‐5p level was significantly down‐regulated in RCC tissues compared with that in adjacent normal tissues. Moreover, we detected the miR‐30d‐5p expression levels in three RCC cell lines (786‐O, ACHN and Caki‐1) and human normal kidney cell line HK‐2. As shown in Fig. 1C, miR‐30d‐5p level was remarkably down‐regulated in all RCC cell lines compared with HK‐2 cells. Among the RCC cells, 786‐O and ACHN cells presented the relatively lower miR‐30d‐5p expression level, and thus were selected for subsequent experiments.

**Fig 1:** miR‐30d‐5p is elevated in RCC cancer tissues and cell lines. (A, B) The expression of miR‐30d‐5p in the cancer tissues and paired normal tissues of 25 patients with RCC. Differences between two groups were assessed by Student's *t*‐test. (C) The expression of miR‐30d‐5p in HK2 and RCC cells (786‐O, ACHN and Caki‐1). Differences among more than two groups were evaluated by one‐way ANOVA, followed by Dunnett's test. Data are presented as mean ± SD of three independent experiments. **P < 0.01, ***P < 0.001, compared with HK‐2.

### miR‐30d‐5p overexpression suppressed cell proliferation and cell‐cycle G1/S transition in RCC cells

Next, we investigated the influence of miR‐30d‐5p on RCC cell proliferation by performing gain‐of‐function assays. The qRT‐PCR results first showed that miR‐30d‐5p mimics transfection significantly elevated the expression of miR‐30d‐5p in both 786‐O and ACHN cells, in comparison with miR‐NC transfection (Fig. 2A). CCK‐8 assay indicated that the proliferation ability of 786‐O and ACHN cells was obviously suppressed after miR‐30d‐5p overexpression (Fig. 2B). Cell growth was closely associated with cell‐cycle progression. We thus analyzed the effects of miR‐30d‐5p overexpression on cell‐cycle distribution in RCC cells. As depicted in Fig. 2C, the percentage of cells at G0/G1 phase was significantly increased; accordingly, cells at S phase were decreased in both 786‐O and ACHN cells after transfection with miR‐30d‐5p mimics compared with miR‐NC transfection. These data suggested that miR‐30d‐5p had a suppressive effect on cell proliferation and cell‐cycle G1/S transition in RCC cells.

**Fig 2:** Effects of miR‐30d‐5p overexpression on cell proliferation and cell‐cycle G1/S transition in RCC cells. 786‐O and ACHN cells were transfected with miR‐30d‐5p mimics or miR‐NC, respectively, for 48 h. (A) The expression of miR‐30d‐5p was determined using qRT‐PCR in transfected 786‐O and ACHN cells. (B) CCK‐8 assay was performed to analyze cell proliferation ability in transfected 786‐O and ACHN cells. (C) The percentage of cells at G0/G1, S and G2/M phases was determined in transfected 786‐O and ACHN cells using flow cytometry with PI staining. Differences between two groups were assessed by Student's *t*‐test. Data are presented as mean ± SD of three independent experiments. **P < 0.01, ***P < 0.001, compared with miR‐NC.

### miR‐30d‐5p overexpression promoted cell apoptosis and inhibited autophagy in RCC cells

In addition to cell‐cycle progression, apoptosis and autophagy have an important role in cell growth, development and the maintenance of cell homeostasis. We subsequently assessed the effects of miR‐30d‐5p on cell apoptosis and autophagy in RCC cells. As shown in Fig. 3A, the total apoptotic rate was significantly elevated after miR‐30d‐5p overexpression in 786‐O and ACHN cells. The immunofluorescence staining indicated that LC3B was decreased in the miR‐30d‐5p mimics group compared with the miR‐NC group in 786‐O and ACHN cells (Fig. 3B).

**Fig 3:** Effects of miR‐30d‐5p overexpression on cell apoptosis and autophagy in RCC cells. 786‐O and ACHN cells were transfected with miR‐30d‐5p mimics or miR‐NC, respectively, for 48 h. (A) Apoptotic rate was measured in transfected 786‐O and ACHN cells using flow cytometry with Annexin V/PI double staining. Differences between two groups were assessed by Student's *t*‐test. Data are presented as mean ± SD of three independent experiments. ***P < 0.001, compared with miR‐NC. (B) Immunofluorescence of LC3B was detected in transfected 786‐O and ACHN cells. Scale bars, 75 µm.

### ATG5 was a direct target of miR‐30d‐5p in RCC cells

To the best of our knowledge, miRNAs influence the biological processes by regulating the downstream target gene via binding its 3′ UTR. Here, bioinformatics analysis prediction showed that the 3ʹ UTR of ATG5 contained a complementary site for the seed region of miR‐30d‐5p (Fig. 4A). Luciferase reporter assay was performed to validate the association between miR‐30d‐5p and ATG5 in two RCC cells. The results showed that the luciferase activity driven by the WT ATG5, but not MUT ATG5, was significantly decreased after miR‐30d‐5p mimics transfection compared with miR‐NC transfection in 786‐O (Fig. 4B) and ACHN (Fig. 4C) cells. Moreover, we explored whether miR‐30d‐5p could directly regulate ATG5 expression. The results indicated that both the mRNA (Fig. 4D) and protein (Fig. 4E) levels of ATG5 were significantly down‐regulated in 786‐O and ACHN cells after miR‐30d‐5p mimics transfection compared with miR‐NC transfection. Results from RNA pull‐down showed that ATG5 was pulled down by miR‐30d‐5p, whereas miR‐30d‐5p‐MUT with mutated binding site of ATG5 failed to pull down ATG5 in 786‐O (Fig. 4F) and ACHN cells (Fig. 4G), indicating that the recognition of miR‐30d‐5p to ATG5 is in a sequence‐specific manner. In addition, ATG5 mRNA expression levels were increased in the 25 fresh RCC tissue samples relative to those in adjacent tissues (Fig. 4H). Furthermore, we detected a statistically significant inverse correlation between miR‐30d‐5p and ATG5 levels in total RCC tissues by Spearman’s correlation analysis (Fig. 4I). These data suggest that ATG5 as a direct target of miR‐30d‐5p was negatively regulated by miR‐30d‐5p in RCC cells.

**Fig 4:** ATG5 was a direct target of miR‐30d‐5p in RCC cells. (A) Predicting binding sites of miR‐30d‐5p to ATG5 3′ UTR. (B, C) Luciferase reporter assay showed that reporter activity was reduced by ~50% after transfection of the WT ATG5 3ʹ UTR reporter and miR‐30d‐5p mimics in 786‐O and ACHN cells. The mRNA (D) and protein (E) levels of ATG5 were determined in 786‐O and ACHN cells after miR‐30d‐5p mimics or miR‐NC transfection using quantitative RT‐PCR and western blot analysis. **P < 0.01, ***P < 0.001, compared with miR‐NC. (F, G) 786‐O (F) and ACHN (G) cells were transfected with biotinylated WT miR‐30d‐5p (miR‐30d‐5p‐Bio) or biotinylated MUT miR‐30d‐5p (miR‐30d‐5p‐MUT‐Bio) or biotinylated NC (NC‐Bio). Forty‐eight hours after transfection, cells were collected for biotin‐based pull‐down assay. ATG5 expression levels were analyzed by quantitative RT‐PCR. ***P < 0.001, compared with NC‐Bio or miR‐30d‐5p‐MUT‐Bio. Differences between two groups were assessed by Student's *t*‐test. Data are presented as mean ± SD of three independent experiments. (H) The mRNA level of ATG5 was measured in cancer tissues and paired normal tissues in 25 patients with RCC. (I) The expression of miR‐30d‐5p was negatively correlated with ATG5 expression in RCC tissues using Pearson's correlation test.

### Restoration of ATG5 reversed the suppressive effects of miR‐30d‐5p on cell proliferation and autophagy in RCC cells

To determine whether ATG5 could reverse the function of miR‐30d‐5p on cell proliferation and autophagy, we cotransfected miR‐30d‐5p mimics and/or pcDNA3.1‐ATG5 into 786‐O cells. As shown in Fig. 5A, the down‐regulated ATG5 expression induced by miR‐30d‐5p overexpression was obviously attenuated by ATG5 overexpression. As expected, the impaired cell proliferation ability by miR‐30d‐5p mimics + pcDNA3.1 transfection was significantly reversed after cotransfection with miR‐30d‐5p mimics and pcDNA3.1‐ATG5 (Fig. 5B). Flow cytometry analysis further confirmed that ATG5 overexpression reversed the function of miR‐30d‐5p mimics on the cell‐cycle G1/S transition (Fig. 5C) and apoptosis (Fig. 5D) of 786‐O cells. In addition, immunofluorescence staining of LC3B showed that the suppressive effects of miR‐30d‐5p overexpression on autophagy were notably abolished by ATG5 overexpression (Fig. 5E). Taken together, these data demonstrated that miR‐30d‐5p could suppress RCC cell proliferation and autophagy by targeting ATG5.

**Fig 5:** Restoration of ATG5 reversed the suppressive effects of miR‐30d‐5p on cell proliferation and autophagy in RCC cells. 786‐O cells were cotransfected with miR‐30d‐5p mimics and/or pcDNA3.1‐ATG5. (A) Western blot analysis of ATG5 protein in transfected 786‐O cells. (B) CCK‐8 assay was performed to analyze cell proliferation ability in transfected 786‐O cells. (C) The percentage of cells at G0/G1, S and G2/M phase was determined in transfected 786‐O cells using flow cytometry with PI staining. (D) Apoptotic rate was measured in transfected 786‐O cells using flow cytometry with Annexin V/PI double staining. Differences among more than two groups were evaluated by one‐way ANOVA, followed by Tukey's test. Data are presented as mean ± SD of three independent experiments. ***P < 0.001, compared with miR‐NC + pcDNA3.1; ^#^ *P* < 0.05, ^##^ *P* < 0.01, compared with miR‐30d‐5p mimics + pcDNA3.1. (E) Immunofluorescence of LC3B was detected in transfected 786‐O cells. Scale bars, 75 µm.

### The regulatory role of miR‐30d‐5p on apoptosis and autophagy‐associated proteins was abolished by ATG overexpression

To better understand the reliance of miR‐30d‐5p on ATG5 for modulation of apoptosis and autophagy of RCC cells, we investigated the expression of apoptosis and autophagy‐related proteins by western blot analysis. As shown in Fig. 6A, miR‐30d‐5p mimics transfection decreased the levels of LC3B‐II/I and Beclin‐1, whereas p62, p21 and Bad expression was up‐regulated in 786‐O cells compared with miR‐NC transfection. Meanwhile, we observed that the regulatory role of miR‐30d‐5p overexpression on the earlier protein expression was remarkably reversed by cotransfection with miR‐30d‐5p mimics and pcDNA3.1‐ATG5 (Fig. 6B). These results further confirmed that ATG5 was a direct target of miR‐30d‐5p in regulating RCC cell apoptosis and autophagy.

**Fig 6:** The regulatory role of miR‐30d‐5p on apoptosis and autophagy‐associated proteins was abolished by ATG overexpression. (A) The expressions of LC3B‐I, LC3B‐II, Beclin‐1, p62, p21 and Bad were measured in 786‐O cells after transfection with miR‐30d‐5p mimics or miR‐NC. Differences between two groups were assessed by Student's *t*‐test. **P < 0.01, ***P < 0.001, compared with miR‐NC. (B) The expressions of LC3B‐I, LC3B‐II, Beclin‐1, p62, p21 and Bad were measured in 786‐O cells after cotransfection with miR‐30d‐5p mimics and pcDNA3.1‐ATG5. Differences among more than two groups were evaluated by one‐way ANOVA, followed by Tukey's test. *P < 0.05, **P < 0.01, ***P < 0.001, compared with miR‐NC + pcDNA3.1; ^##^ *P* < 0.01, ^###^ *P* < 0.001, compared with miR‐30d‐5p mimics + pcDNA3.1. Data are presented as mean ± SD of three independent experiments. GAPDH, glyceraldehyde‐3 phosphate dehydrogenase.

## Discussion

Here, we found that miR‐30d‐5p was significantly down‐regulated in RCC tissues and cell lines compared with corresponding controls. Further functional experiments showed that overexpression of miR‐30d‐5p remarkably suppressed cell proliferation and cell‐cycle G1/S transition in two RCC cell lines (786‐O and ACHN). Consistent with our data, the suppressive role of miR‐30d‐5p on tumor cell proliferation has been revealed in non‐small cell lung cancer [11], gallbladder carcinoma [12], prostate cancer [13] and colon cancer [21]. In addition, we observed that overexpression of miR‐30d‐5p promoted cell apoptosis by up‐regulating Bad expression in RCC cells. In line with our data, overexpression of miR‐30d‐5p reduced proliferation and induced the ovarian granulosa cell apoptosis by targeting Smad2 [22].

Autophagy plays dual roles in tumorigenesis by suppressing the growth of cancer cells at early stage or promoting rapid growth of malignant cells at later stages [23, 24. Previous studies have illustrated the vital role of autophagy in the growth and progression of RCC. For instance, LC3B‐mediated autophagy promotes the growth of von Hippel–Lindau‐negative RCC tumors [25]. The activation of autophagy under starvation conditions by TRPM3 overexpression caused the accelerating growth of von Hippel–Lindau‐negative RCC cells [26]. In our study, we observed that overexpression of miR‐30d‐5p inhibited autophagy by down‐regulating LC3BII/I and Beclin‐1, but up‐regulating p62 expression. LC3B staining is usually associated with high levels of autophagy [27]. It has been suggested that p62 plays a crucial role in autophagosome for autophagic degradation [28], which was accumulated during inhibition of autophagy and decreased during activation of autophagy [29]. Moreover, the study further supported our data that Lotze *et al*. [30] demonstrated that pharmacological inhibition of autophagy will be a novel approach for the treatment of RCC.

More importantly, we demonstrated that ATG5 was a direct target of miR‐30d‐5p in RCC cells. In addition, it was verified that miR‐30d‐5p promoted cell apoptosis and repressed autophagy by targeting ATG5 through performing rescue experiments. As shown by a large number of studies, inhibition of autophagy, accompanied with decreased expression of ATG5, has been an effective strategy to overcome acquired resistance in non‐small cell lung cancer [31], hepatocellular carcinoma [32] and breast cancer [33]. Furthermore, ATG5 has been identified as miR‐30b in hepatocellular carcinoma [34], osteosarcoma [35] and gastric cancer [36]. Considering the potential targeted regulation between miR‐30d and ATG5 in the earlier described tumors, we thus speculated that ATG5 was a downstream direct regulator participating in miR‐30d‐5p‐inducing decreased proliferation and autophagy in RCC cells.

In summary, our study for the first time demonstrated that miR‐30d‐5p inhibited cell proliferation and autophagy, as well as induced cell‐cycle arrest and apoptosis by targeting ATG5 in RCC cells *in vitro*. Our data suggest that miR‐30d‐5p has high potential as a tumor suppressor that could be exploited in the development of novel anticancer therapeutics.

## Conflict of interest

The authors declare no conflict of interest.

## Author contributions

L. Lei conceived and designed the project. L. Liang and ZY performed the study and acquired the data. QD, YJ and YC analyzed and interpreted the data. YS wrote and revised the paper. All authors read and approved the final manuscript.

## Data Availability

Data are available on request from the corresponding author.
